The article "Hybrid Deep Feature Fusion of 2D CNN and 3D CNN for Vestibule Segmentation from CT Images" was published in 2022. Journal: Comput Math Methods Med.

# Hybrid Deep Feature Fusion of 2D CNN and 3D CNN for Vestibule Segmentation from CT Images

**DOI:** 10.1155/2022/6557593

**Published:** 2022-04-12

**Authors:** Ruicong Zhang, Li Zhuo, Meijuan Chen, Hongxia Yin, Xiaoguang Li, Zhenchang Wang

**Affiliations:** ^1^Faculty of Information Technology, Beijing University of Technology, Beijing 100124, China; ^2^Department of Radiology, Beijing Friendship Hospital, Capital Medical University, Beijing 100050, China

## Abstract

The accurate vestibule segmentation from CT images is essential to the quantitative analysis of the anatomical structure of the ear. However, it is a challenging task due to the tiny size, blur boundary, and drastic variations in shape and size. In this paper, according to the specific characteristics and segmentation requirements of the vestibule, a vestibule segmentation network with a hybrid deep feature fusion of 2D CNN and 3D CNN is proposed. First, a 2D CNN is designed to extract the intraslice features through multiple deep feature fusion strategies, including a convolutional feature fusion strategy for different receptive fields, a feature channel fusion strategy based on channel attention mechanism, and an encoder-decoder feature fusion strategy. Next, a 3D DenseUNet is designed to extract the interslice features. Finally, a hybrid feature fusion module is proposed to fuse the intraslice and interslice features to effectively exploit the context information, thus achieving the accurate segmentation of the vestibule structure. At present, there is no publicly available dataset for vestibule segmentation. Therefore, the proposed segmentation method is validated on two self-established datasets, namely, VestibuleDataSet and IEBL-DataSet. It has been compared with several state-of-the-art methods on the datasets, including the general DeeplabV3+ method and specific 3D DSD vestibule segmentation method. The experimental results show that our proposed method can achieve superior segmentation accuracy.

## 1. Introduction

The vestibule is one of the important organs in the inner ear, located between the cochlea and the semicircular canal. The accurate segmentation of the vestibule is fundamental to the quantitative analysis of the anatomical structure of the ear, which is significant for the clinical diagnosis of ear diseases [1, 2]. As shown in Figure 1, the vestibule is highlighted in blue. It can be seen that it is relatively small. Although the existing image semantic segmentation networks based on deep learning, such as DeepLab series, have achieved high segmentation accuracy, they cannot work well when applied to the vestibule segmentation task, due to the following facts: (i) the vestibule has a precise structure with very few voxels, and the boundary between the cochlea and semicircular canals is not clear, as shown in Figure 1; (ii) the sample data is difficult to label because it is time-consuming and due to labor cost.

The article "Hybrid Deep Feature Fusion of 2D CNN and 3D CNN for Vestibule Segmentation from CT Images" was published in 2022. Journal: Comput Math Methods Med.

Medical image has unique characteristics that are different from natural image. To obtain good segmentation performance, it is necessary to design a specific network architecture according to the characteristics of medical images and the requirements of the segmentation task. In recent years, 3D CNN has gradually attracted researcher's attention in medical image segmentation tasks. Since most of medical data such as CT and MRI images exist in the form of 3D volume data, the use of 3D CNN can better mine the inherent correlation of the data. Therefore, some researchers applied 3D CNN in medical image segmentation tasks. Besides, it was also exploited in other segmentation tasks and achieved good performance, such as foreground segmentation [3] and moving object segmentation [4].

At present, the segmentation methods are usually designed for specific medical image segmentation tasks. There are relatively few methods for vestibule segmentation. In [5], to solve the segmentation problem of sophisticated and small organs of the ears, a novel 3D Deep Supervised Dense Network (3D DSD) has been proposed. The authors adopted a dense connection structure and proposed a 3D multipooling feature fusion strategy to segment nine different ear organs simultaneously, including the vestibule. However, it is hard to train the 3D DSD network, and the segmentation performance is not too high. In our previous research work, we proposed a 2D CNN for the vestibule segmentation, which integrates multiple deep feature fusion strategies [6]. Since the segmentation method based on 2D CNN cannot make good use of the interslice correlations, the segmentation performance is to be improved.

In this paper, we design a vestibule segmentation network for CT images. The network extracts the intraslice features with 2D CNN and interslice features with 3D CNN, respectively. Then, the two kinds of features are fused with a hybrid feature fusion module to realize the accurate segmentation of the vestibule. The proposed segmentation method is demonstrated on two self-established datasets, namely, VestibuleDataSet and IEBL-DataSet. The experimental results show that, compared with several state-of-the-art segmentation methods, our proposed method can achieve superior segmentation accuracy.

The rest of this paper is organized as follows.  Section 2 provides a detailed presentation of the proposed vestibule segmentation network, and Section 3 describes the experimental results and analysis in detail. The conclusions are drawn in Section 4.

The article "Hybrid Deep Feature Fusion of 2D CNN and 3D CNN for Vestibule Segmentation from CT Images" was published in 2022. Journal: Comput Math Methods Med.

## 2. Proposed Vestibule Segmentation Network

A proposed vestibule segmentation network is shown in Figure 2, in which a 2D CNN is designed to extract the intraslice features, and a 3D DenseUNet to extract the interslice features. And then, the two kinds of features are fused through a hybrid feature fusion module. The whole network framework can be divided into three key components, 2D CNN, 3D DenseUNet, and hybrid feature fusion module, which will be introduced in detail.

### 2.1. 2D CNN with Multiple Deep Feature Fusion Strategies

In our previous research work [6], we designed a 2D CNN vestibule segmentation network with multiple deep feature fusion strategies. The network adopts the basic framework of encoder-decoder [7–9], as shown in Figure 3. Three feature fusion strategies are integrated to realize the accurate vestibule segmentation, namely, (i) a convolution feature fusion strategy for different receptive fields, (ii) a feature channel fusion strategy based on channel attention mechanism, and (iii) an encoder-decoder feature fusion strategy.

In this paper, this method is improved to extract the intraslice features. As shown in Figure 3, the main improvements are as follows: (1) To extract the deep features better, we use five layers of block in the encoder and decoder, respectively. (2) Downblock is elaborately designed, which is composed of convolution layer, SEblock layer, batch norm layer, and ReLU layer. Max pooling is used in Downblock1 and average pooling in Downblock2~Downblock4, respectively. (3) SEblock is removed from the decoder. And cascading operation is used for the connection between the encoder and decoder. Experimental results demonstrate that the above improvements can effectively improve the segmentation performance of 2D CNN.

### 2.2. 3D DenseUNet Structure

To deal with the dramatic changes among different slices of the vestibule, in this paper, DenseNet-BC and U-Net are integrated together to obtain a 3D DenseUNet network, which is used to extract the interslice features. DenseNet adopts a feed-forward way to connect the layers. For each layer, all the feature maps of the previous layer are used as input. This connection manner can strengthen the transfer of features, and the information of different scales can be fully utilized. In addition, it also has fewer parameters, making the network easier to train. The network structure using the bottleneck layer and the transition layer is named as DenseNet-BC.

In the encoder part, the DenseNet architecture is adopted. Due to the high memory consumption of 3D convolution and the limitation of GPU memory, we reduce the number of convolution layers of each dense block to be half of the original DenseNet-121 and set the growth rate *K* as 32. The feature size of the input is 224 × 224 × 8, and the feature size of the output after downsampling is 7 × 7 × 2. The parameters of each layer of the decoder are shown in Table 1. The UNet long-range connection links the encoder and the decoder, and the feature size of the output after upsampling is 224 × 224 × 8.

The article "Hybrid Deep Feature Fusion of 2D CNN and 3D CNN for Vestibule Segmentation from CT Images" was published in 2022. Journal: Comput Math Methods Med.

### 2.3. Hybrid Feature Fusion Module

In order to fuse the features extracted by 2D CNN and 3D DenseUNet, a hybrid feature fusion (HFF) module is designed in this paper. HFF is composed of convolution layer, dropout layer, BN layer, and ReLU layer, as shown in Figure 4.

The output feature of 2D CNN is represented by the output of upblock 5; the feature size is 224 × 224. The output features of 3D DenseUNet are represented by the output of upsampling layer 5, and the feature size is 224 × 224 × 8. Before fusion, it is necessary to ensure that the size of the feature maps is the same. The function *ƒ* represents the conversion of a 3D volume to two adjacent 2D slices, and the function *ƒ*^−1^ represents the inverse conversion of two adjacent 2D slices to a 3D volume. The specific conversion process is shown in Figure 2. Firstly, the output feature 8 × 224 × 224 × 64 of the 2D CNN is converted into a volume form of 224 × 224 × 8 × 64 through *ƒ*^−1^. 3D DenseUNet takes the original 3D images and the images segmented by the 2D network as input by concatenating it, which can reduce the optimization burden of the 3D network and avoid learning useless features. Then, the 2D CNN features and 3D DenseUNet features are cascaded to obtain 224 × 224 × 8 × 64 features and sent to HFF. The output of the HFF module is 224 × 224 × 8 × 2.

### 2.4. Loss Function

The cross-entropy loss function compares the predicted value with the ground truth pixel by pixel. This function has the same weights for each category, so it is very vulnerable to the category imbalance. We use the weighted cross-entropy loss function to train the network model, which assigns a weight factor for each category, as shown in Equation (1), to solve the problem of category imbalance.

(1) $$\begin{array}{c} L_{\text{Weighted Cross}‐\text{Entropy}}\left(y,y\_\text{pred}\right)=-\frac{1}{n}\overset{n}{\underset{i=1}{\sum }}\overset{2}{\underset{c=1}{\sum }}w_{i}^{c}y_{i}^{c}\log y\_\text{pre}{\text{d}}_{i}^{c}, \end{array}$$

where *y* is ground truth, *y*_pred is the predicted value, *c* is the number of categories, *w*_*i*_ is the weight factor of *i*-th category, and *n* is the total number of data samples.

## 3. Experimental Results and Analysis

### 3.1. Datasets and Evaluation Metrics

Since there is currently no publicly available dataset for ear segmentation, we established a vestibule segmentation dataset, namely, VestibuleDataSet, and an inner ear bone labyrinth segmentation dataset, namely, IEBL-DataSet. All CT images were collected from Beijing Friendship Hospital affiliated with Capital Medical University. According to actual application requirements, we invited radiologists with rich clinical experience to label the data in three dimensions. The collected CT images were all scanned with a Phillips 64-slice spiral CT scanner on the CT cross-section of the temporal bone. The specific scanning parameters are as follows: tube current is 300 mAs, tube voltage is 120/140 kV, FOV is 14 cm × 14 cm ~ 18 cm × 18 cm, the layer thickness is 0.625 mm/0.67 mm, the resolution is 512 × 512, the pitch is 0.32 mm, window width is 4000 HU, and window level is 700 HU. VestibuleDataSet is divided into three parts: training set (82 samples), validation set (10 samples), and test set (10 samples).

The article "Hybrid Deep Feature Fusion of 2D CNN and 3D CNN for Vestibule Segmentation from CT Images" was published in 2022. Journal: Comput Math Methods Med.

All of the data samples in IEBL-DataSet were collected using ultrahigh resolution CT scanner, which was developed elaborately for scanning the ears. Each case of the UHRCT dataset contains image data from the top of the rock cone to the stylomastoid on both sides. Among them, the single-sided data axis plane contains 370 images. The scanning parameters are as follows: receptive field of 65 mm × 65 mm, axial resolution of 650 × 650, tube voltage of 100 kV, tube current of 3.5 mA, and pixel spacing, layer thickness, and layer spacing are all 0.1 mm. IEBL-DataSet contains 68 samples. They are divided into three parts: training set (47 samples), validation set (7 samples), and test set (14 samples).

In order to comprehensively evaluate the segmentation performance, we use three commonly used evaluation metrics, namely, Dice similarity coefficient (DSC), average symmetric surface distance (ASD) [10], and average Hausdorff distance (AVD) [11].

### 3.2. Parameter Setting

The method proposed in this paper was implemented and tested on the Keras platform with two Nvidia Geforce GTX 1080Ti 11GB GPUs. In the training phase, the SGD [12] optimizer was used. The initial learning rate, weight decay factor, and momentum were set as 0.008, 0.00005, and 0.9, respectively. Small-scale scaling operations and random flip operations with a threshold range of 0.8 to 1.2 were used to expand the number of the data samples, which can effectively avoid overfitting in the training process. It took about 24 hours and 72 hours to train the 2D CNN and 3D DenseUNet models, respectively.

### 3.3. Comparisons with the State-of-the-Art Segmentation Methods on VestibuleDataSet

To verify the effectiveness of the segmentation method proposed in this paper, we compared it with several state-of-the-art segmentation methods, including DeeplabV3 + [13], 2D CNN based on multiple deep feature fusion strategies [6], and 3D DSD [5]. DeeplabV3+ is the most representative semantic segmentation method for natural images with better segmentation performance. 2D CNN based on multiple deep feature fusion strategies is a network dedicated to the vestibule segmentation proposed in our previous research work. 3D-DSD is a network dedicated to temporal bone segmentation, including vestibule segmentation. All network models were trained on VestibuleDataSet. The experimental results are shown in Table 2.

The article "Hybrid Deep Feature Fusion of 2D CNN and 3D CNN for Vestibule Segmentation from CT Images" was published in 2022. Journal: Comput Math Methods Med.

It can be seen from Table 2 that, compared with the 2D CNN and 3D DSD segmentation methods, the mean DSC of the proposed method increases by 2.38% and 3.89%, respectively, reaching 87.00%. Compared with the 3D DSD segmentation method, although our proposed method has a larger mean ASD value, the mean AVD value is smaller, and the mean DSC value is much higher. It demonstrates that our proposed method can achieve better segmentation performance. In addition, all the segmentation performances of 2D CNN, 3D DSD, and our proposed segmentation method are better than that of the DeeplabV3+ segmentation method. It means that the specific network designed according to the characteristics of the vestibule can achieve better segmentation performance than the general network.

Figure 5 shows 4 the visualized segmentation results using our proposed method on the test set. The result is a subjective visualization of the axis position. To show the results more clearly, we expanded the segmentation results by 3 times. The green area represents the ground truth, the red area represents the segmentation results, and the yellow area represents the overlap areas between the ground truth and the prediction results. The larger the overlap areas, the better the segmentation results. It can be seen from Figure 5 that our proposed method can segment the vestibule well. On the whole, oversegmentation is more serious than undersegmentation. This is because the vestibule structure is tiny, the boundary is not clear, and oversegmentation often occurs.

Figure 6 shows the comparison of the segmentation results using DeeplabV3+, 2D CNN based on multiple deep feature fusion strategies, 3D DSD, and our proposed method. It can be seen from Figure 6 that DeeplabV3+ and 3D DSD have serious undersegmentation problems. The 2D CNN based on multiple deep feature fusion strategies and our proposed method can segment the vestibule accurately. In general, the segmentation results of our proposed method are much closer to the ground truth, which illustrates its superiority over the existing segmentation methods.

The article "Hybrid Deep Feature Fusion of 2D CNN and 3D CNN for Vestibule Segmentation from CT Images" was published in 2022. Journal: Comput Math Methods Med.

### 3.4. Comparisons with the State-of-the-Art Segmentation Methods on IEBL-DataSet

To demonstrate the effectiveness of the proposed method, we further conducted comparison experiments on another self-established dataset for inner ear bone labyrinth segmentation, namely, IEBL-DataSet. The comparison methods include DeeplabV3+ [13], 3D DSD [5], and 2D CNN [6]. The comparison results using different segmentation methods are shown in Table 3.

It can be seen that our proposed method can obtain the highest accuracy, reaching 88.93 of DSC, 1.69%, 0.98%, and 1.56% higher than those of DeeplabV3+, 3D DSD, and 2D CNN, respectively. ASD are up to 0.41, 0.25, and 0.33 lower than those of DeeplabV3+ and 2D CNN, respectively.

Figure 7 shows the visualized segmentation results by using different methods. The yellow area shown in Figure 7(a) is the ground truth. Green and pink areas represent the undersegmented and oversegmented parts, respectively. It can be seen that other segmentation methods are easily affected by the surrounding pixels, resulting in oversegmentation or undersegmentation. Our segmentation method can obtain more accurate segmentation results. All the above results show that our method has good robustness and generalization capability.

### 3.5. The Parameter Scale of the Proposed Method

Table 4 shows the parameter scale of our proposed method and comparison methods. It can be seen that the parameter scale of the proposed method is much higher than those of the comparison methods, since it fuses the deep features of 2D CNN and 3D CNN. And the average inference time for a 224 × 224 image is about 0.02 second with the aid of GPU accelerator. It means that our proposed method can improve the segmentation accuracy, but at the cost of the computational complexity of the model. In our future work, it is also necessary to reduce the consumption of computing resources while maintaining the segmentation accuracy.

### 3.6. Ablation Studies

The network architecture proposed in this paper consists of three key components, i.e., 2D CNN, 3D DenseUNet, and hybrid feature fusion module. To evaluate the effect of different modules on the overall segmentation performance, we conducted ablation studies.  Table 5 shows the segmentation results obtained by using different modules, in which A indicates that only 2D CNN is used, A+B indicates 2D CNN is fused with the original 3D volume and then sent to 3D DenseUNet for training, and A+B+C indicates the proposed method.

The article "Hybrid Deep Feature Fusion of 2D CNN and 3D CNN for Vestibule Segmentation from CT Images" was published in 2022. Journal: Comput Math Methods Med.

It can be seen from Table 5 that (1) compared with the original 2D CNN with multiple deep feature fusion strategies, the improved 2D CNN increase the segmentation accuracy by 1.08%. It demonstrates the effectiveness of the improved 2D CNN method. (2) Each module leads to a significant improvement in segmentation performance, and when the three modules are used together, the highest segmentation performance can be obtained. The reason is that 2D CNN can extract the intraslice features, and 3D CNN can extract the interslice features, and the hybrid feature fusion module can help to make full use of the intra- and interslice features, thus achieving better segmentation performance.

## 4. Conclusions

According to the specific structural characteristics and segmentation requirements of the vestibule, we design a network architecture through hybrid deep feature fusion of 2D CNN and 3D CNN. First, a 2D CNN based on multiple deep feature fusion strategies is used to extract the intraslice features and 3D DenseUNet to extract the interslice features. Then, a hybrid feature fusion module is designed to fuse the two kinds of features. Experimental results show that our proposed segmentation network can achieve a higher segmentation accuracy and good generalization ability. In future work, we will design an efficient CNN network to further improve the segmentation accuracy with lower computational complexity.

## Figures and Tables

**Figure 1:** An example of the vestibule structure from CT image. The vestibule is highlighted in blue.

**Figure 2:** The framework of the proposed vestibule segmentation network.

**Figure 3:** The framework of 2D CNN.

**Figure 4:** The framework of HFF.

**Figure 5:** Example of segmentation results by using our proposed method.

**Figure 6:** Comparison of segmentation results of several methods.

**Figure 7:** The visualization comparison results of IEBL-DataSet. (a) The ground truth. (b) The segmented results of our proposed method. (c–e) The segmentation results obtained by using the three comparison methods, respectively.

**Table 1:** Parameter setting of each module of 3D DenseUNet.

Block	Feature size	Convolution layer
Input	224 × 224 × 8	—
Convolution 1	112 × 112 × 4	7 × 7 × 7 × 96 conv
Pooling	56 × 56 × 2	3 × 3 × 3 max pooling
Dense block 1	56 × 56 × 2	(1 × 1 × 1 × 128 conv) × 3 (3 × 3 × 3 × 32 conv) × 3
Transition layer 1	28 × 28 × 2	1 × 1 × 1 conv 2 × 2 × 1 average pooling
Dense block 2	28 × 28 × 2	(1 × 1 × 1 × 128 conv) × 4 (3 × 3 × 3 × 32 conv) × 4
Transition layer 2	14 × 14 × 2	1 × 1 × 1 conv 2 × 2 × 1 average pooling
Dense block 3	14 × 14 × 2	(1 × 1 × 1 × 128 conv) × 12 (3 × 3 × 3 × 32 conv) × 12
Transition layer 3	7 × 7 × 2	1 × 1 × 1 conv 2 × 2 × 1 average pooling
Dense block 4	7 × 7 × 2	(1 × 1 × 1 × 128 conv) × 8 (3 × 3 × 3 × 32 conv) × 8
Upsampling layer 1	7 × 7 × 2	2 × 2 × 1 × 504 upconv
Sum with dense block 3	14 × 14 × 2	—
Upsampling layer 2	14 × 14 × 2	2 × 2 × 1 × 224 upconv
Sum with dense block 2	28 × 28 × 2	—
Upsampling layer 3	28 × 28 × 2	2 × 2 × 1 × 192 upconv
Sum with dense block 1	56 × 56 × 2	—
Upsampling layer 4	56 × 56 × 2	2 × 2 × 2 × 96 upconv
Sum with convolution 1	112 × 112 × 4	—
Upsampling layer 5	224 × 224 × 8	2 × 2 × 2 × 64 upconv
Output	224 × 224 × 8	1 × 1 × 1 × 3 conv

The article "Hybrid Deep Feature Fusion of 2D CNN and 3D CNN for Vestibule Segmentation from CT Images" was published in 2022. Journal: Comput Math Methods Med.

**Table 2:** Comparison results of segmentation performance by using our proposed method and other methods.

Method	DSC (%)	ASD (mm)	AVD (mm)
DeeplabV3+ [13]	76.36	0.38	6.95
2D CNN [6]	84.62	0.23	0.64
3D DSD [5]	83.11	0.19	0.27
Ours	87.00	0.21	0.24

**Table 3:** Comparison results using different segmentation methods on the IEBL-DataSet.

Method	DSC (%)	ASD (mm)
DeeplabV3+ [13]	87.46	0.66
3D DSD [5]	88.17	0.39
2D CNN [6]	87.59	0.74
Ours	89.15	0.41

**Table 4:** Parameter scale of different methods.

Method	Parameter scale
UNet [14]	7.77 MB
DeeplabV3+ [13]	41 MB
3D DSD [5]	9.86 MB
Ours	95.4 MB

**Table 5:** Effect of different modules on segmentation performance.

Method	DSC (%)	ASD (mm)	AVD (mm)
A	85.70	0.24	1.80
A+B	86.65	0.22	0.25
A+B+C	87.00	0.21	0.24

## Data Availability

The copyright of the data used in this paper belongs to Beijing Friendship Hospital affiliated with Capital Medical University. So it cannot be disclosed without authorization.
